# Acute Toxicity and Gastroprotection Studies of a New Schiff Base Derived Manganese (II) Complex against HCl/Ethanol-Induced Gastric Ulcerations in Rats

This article has been retracted.

**DOI:** 10.1038/srep26819

**Published:** 2016-05-27

**Authors:** Mohamed Yousif Ibrahim, Najihah Mohd Hashim, Summaya M. Dhiyaaldeen, Mazen M.Jamil Al-Obaidi, Rashd M. El-Ferjani, Hoyam Adam, Bassam Alkotaini, Rami Al Batran, Hapipah Mohd Ali

**Affiliations:** 1 Department of Pharmacy, Faculty of Medicine, University of Malaya 50603 Kuala Lumpur, Malaysia; 2 Department of Chemistry, Faculty of Science, University of Malaya, 50603 Kuala Lumpur, Malaysia; 3 Center for Natural Products and Drug Discovery (CENAR), University of Malaya, Kuala Lumpur, Malaysia; 4 Department of Microbiology, Faculty of medicine, University of Duhok, 78 Kurdistan, Iraq; 5 Department of Biomedical Science, Faculty of Medicine, University of Malaya, 50603 Kuala Lumpur, Malaysia; 6 Department of Chemistry, Faculty of Science, University of Benghazi, 1308 Benghazi, Libya; 7 School of Pharmacy, Ahfad University for Women (AUW), 167 Omdurman, Sudan; 8 Department of Chemical Engineering, Faculty of Engineering, Chungbuk National University, Cheongju, Chungbuk 28644, Republic of Korea; 9 Institute of Research Management & Monitoring, Deputy Vice Chancellor (Research & Innovation), University of Malaya, 50603 Kuala Lumpur, Malaysia

## Abstract

Manganese is a crucial element for health. In this study, the gastroprotective efficacy *of* Mn (II) complex (MDLA) against acidified ethanol (HCl/Ethanol)-induced gastric ulceration in rats was evaluated. The animals were distributed into 5 groups. Groups 1 and 2 received carboxymethylcellulose (CMC), group 3 was pretreated with omeprazole, and groups 4 and 5 were given 10 and 20 mg/kg of MDLA, respectively. After one hour, CMC and HCl/Ethanol were given to groups 2–5 whilst the animals in group 1 were ingested with CMC. After sacrifice, gastric lesions were evaluated by wall mucus, gross appearance, histology, antioxidant enzymes and immunohistochemistry. Group 2 displayed severe gastric damage with a significant reduction in wall mucus. Conversely, gastric lesions were reduced in groups 3–5 by 85.72%, 56.51% and 65.93%, respectively. The rats in groups 3–5 showed up-regulation of heat shock protein 70 (Hsp70) with down-regulation of Bcl-2-associated protein x (Bax). Pretreatment with omeprazole or MDLA led to an increase in the uptake of Periodic Acid Schiff (PAS) stain in the glandular part of the gastric tissue, raised levels of prostaglandin E2 (PGE_2_) and superoxide dismutase (SOD), and a reduction in malondialdehyde (MDA) concentrations. These results suggested the gastroprotective action of Mn (II) complex.

Gastric ulcer is the most common gastrointestinal pathology and affects approximately 10–15% of the world’s population; its prevalence rate is associated with age and sex, as well as lifestyle^1^. This disease is characterized by mucosal impairment in the gastric accompanied by stomachache, vomiting, loss of appetite and weight, and hemorrhage and perforation. The progression of gastric ulceration is attributed to infection by *Helicobacter pylori*, overuse of non-steroidal anti-inflammatory drugs (NSAIDs) and immunosuppressive treatments, as well as alcohol abuse and smoking^2^.

Although, the gastrointestinal tract is commonly exposed to countless microbes and harmful substances as well as food antigens, the surface of gastric mucosa is protected by a distinct barrier mechanism. Certain immune reactions to these antigens enhance the mucosal defense system to sustain homeostasis of the digestive system^3^. The inability of the defensive factors, such as bicarbonate secretion, mucus-bicarbonate barrier, surface active phospholipids, prostaglandins (PGs), mucosal microcirculation, cell regeneration, endogenous antioxidants, endogenous nitric oxide and certain growth factors to adequately suppress the aggressive factors, which comprise gastric acid and pepsin secretion, *Helicobacter pylori*, refluxed bile, release of leukotrienes and reactive oxygen species (ROS), result in stomach injury^4^.

Even though developments have been conducted in terms of a cure of gastric ulcerations, the mortality rates are still high^5^. The current medications for the treatment of ulcerations suffer a serious disadvantage as they are accompanied by high decline rates and increasing side effects^6^.

Authentication of the effectiveness and utilization of synthetic agents for the cure of gastric ulceration disease is a promising way to overcome the shortcomings of orthodox medications^7^.

In this respect, Schiff bases are deemed to be a substantial category of organic agents in the field of medicinal chemistry^8^, and the study of new Schiff base complexes accompanied by therapeutic efficacy is attracting the interest of researchers^9^. Schiff bases, along with their transition metal complexes, are multifunctional agents resulting from the reaction of an amino candidate with a carbonyl agent. In addition, they are extensively utilized for industrial objectives and in a wide range of pharmacological applications comprising antifungal, antibacterial, antimalarial, antiproliferative, anti-inflammatory, antiviral, and antipyretic activities^10^.

Manganese (Mn), which is a crucial element for human health and acts as a significant part of the antioxidant system, is found in several enzymes, such as mitochondrial superoxide dismutases, glutamine synthetase, alkaline phosphatase, and arginase^11^. Although surplus Mn^2+^ is poisonous and can result in damage, and lead to a Parkinsonian-like syndrome^12^, lower concentrations can have a defensive effect by decreasing the radical dotOH to yield Mn(OH)^2+ ^13. In addition, manganese-containing superoxide dismutase (Mn-SOD) has attracted specific interest since it enhances the antioxidant properties and contributes to cancer protection^14^.

The present study was performed to study the mechanism of the anti-ulcerogenic effect of the new Mn (II) complex with a Schiff base derived from 4-dimethylaminobenzaldehyde with L-asparagine (MDLA) against acidified ethanol (HCl/Ethanol)-induced gastric ulcers in rats.

## Materials and Methods

### Chemicals, reagents and drugs

All chemicals and reagents were purchased from Sigma (Sigma Aldrich, Germany) and used without further purification. In addition, malondialdehyde (MDA), superoxide dismutase (SOD) and prostaglandin E2 (PGE_2_) Kits were obtained from Cayman Chemical Company (Cayman, USA). Omeprazole was utilized as a reference antiulcer medication and was acquired from the University of Malaya Medical Centre (UMMC) Pharmacy. This medication was prepared as a suspension in 0.5% (w/v) carboxymethylcellulose (CMC) and intragastrically administered to the rats at a dose of 20 mg/kg body weight (5 ml/kg) according to the suggestions of Miranda *et al.*^15^.

### Preparation of the Schiff base

The Schiff base formed from 4-dimethylaminobenzaldehyde and L-asparagine was prepared by adding 25 ml of 4-dimethylaminobenzaldehyde ethanolic solution (1.49, 0.01 mol) to an equal amount of ethanolic solution of L-asparagine (0.01 mol). The mixture was refluxed for two hours. The product that formed was collected by filtration, washed several times with ethanol and recrystallized from hot ethanol^16^.

### Preparation of Schiff base metal complex

The Mn (II) complex (Fig. 1) was prepared by adding 25 ml of ethanolic solution of metal chloride (0.01 mole) with ethanolic solutions of the prepared Schiff base (0.01 mole) followed by the drop-wise addition of aqueous ammonia. The resulting mixture was refluxed for two hours and the metal complex compounds that precipitated out were filtered and then washed repeatedly with hot ethanol until the washing was colorless. The product was air dried over phosphorus penta-oxide^16^. Elemental analysis and spectral characterization for the ligand and its metal complex are presented in Table 1.

### Ethical issues

All the methods were carried out in accordance with the approved guidelines of the Institutional Animal Ethical Committee of the University of Malaya [Ethic certificate no. (PM/27/7/2014/RAB (R)]. Pathogen-free Sprague-Dawley rats with an average body weight of (200–220 g), were provided by the Animal House, Faculty of Medicine, University of Malaya, Kuala Lumpur. The rats were fed a standard diet and tap water *ad libitum,* and were kept separately in cages with wide-mesh wire bottoms to prevent coprophagia throughout the experiment.

### Acute toxicity test and experimental animals

The acute toxicity study was carried out to determine a nontoxic dosage for MDLA. Thirty-six rats (18 male and 18 female) were separately and equally allocated into 3 groups labeled as vehicle (0.5% CMC, 5 ml/kg) or as 500 or 1000 mg/kg of MDLA (5 ml/kg). The animals were deprived of food overnight before treating. Food was withdrawn for an additional 3 to 4 h after treatment. The rats were monitored for 48 hours after the intragastric administration of the MDLA for toxicological signs. Death cases were recorded over a duration of 14 consecutive days. All the rats were killed via an overdose of xylazine and ketamine anesthesia on the 15^th^ day and then histological evaluation and serum analysis were implemented following the standard techniques^17^,^18^.

### Gastric ulcer study and experimental animals

The animals were randomly distributed into 5 groups of 6 rats each in separate cages with wide-mesh wire bottoms to prevent coprophagia during the experiment. Animals were deprived of food for 24 h but allowed free access to drinking water up to 2 hours before conducting the experimentation. The gastric ulceration model was induced using acidified ethanol solution (150 mM Hcl/absolute ethanol) 40: 60 v/v, (Hcl/ethanol solution) based upon a published protocol with some modification^15^. For groups 1 and 2, the vehicle (0.5% CMC) was administered intragastrically. Meanwhile, group 3 received an oral dosage of 20 mg/kg omeprazole in 0.5% CMC (5 ml/kg), and groups 4–5 were administered MDLA at doses of 10 and 20 mg/kg, respectively. These dosages were administered as pre-treatment. One-hour after pre-treatment, the vehicle and acidified ethanol (HCl/Ethanol) were intragastrically administered to group 1 and groups 2–5, respectively. The rats were euthanized (xylazine and ketamine) after 60 min, and their stomach tissues were dissected.

### Determination of gastric volume, pH and mucus in gastric content

The stomachs were removed, opened along the greater curvature, and their contents were placed in labeled tubes and centrifuged at 2000 rpm for 10 min. The pH of the resultant supernatant was recorded using a digital pH meter (PA 200, Marconi S.A, Brazil). Quantitative estimation assay of the gastric mucus was implemented according to the methodology previously reported by Corne *et al.*^19^.

### Macroscopic gastric lesion evaluation

The ulcerative injuries (mm^2^) were investigated using a 10× magnifier lens to assess the formation of ulcerations. The sum of the ulcer area for each animal was calculated and used as the ulcer index (UI). The Inhibition/Gastroprotection percentage (I %) was calculated according to the following formula:

Inhibition percentage (I %) = [(UI control − UI treated) ÷ UI control] × 100%.

### Anti-oxidant activity

#### Preparation of tissue homogenates

Gastric tissue specimens were rinsed thoroughly and then homogenized using a mortar. The homogenized tissues (10% w/v) were prepared in an ice-cold 50 mM phosphate buffer (pH 7.4) comprising a mammalian protease inhibitor cocktail. The homogenates were then centrifuged at 4,000 rpm for 10 minutes (4 °C). The resulting supernatant was employed to quantify the enzymatic activities.

#### Measurement of SOD activity

SOD activity was determined using the method described by Sun *et al.*^20^. The suppression of the photochemical reduction of nitroblue tetrazolium (NBT) to produce blue colored formazan salt in existence of phenazine methosulphate (PMS) besides reduced nicotinamide adenine dinucleotide (NADH) was assessed at 560 nm using n-butanol as blank. SOD activity was expressed as units/mg protein.

#### Measurement of MDA

Tissue malondialdehyde (MDA) (mmol/L) was measured using the previously reported method of Draper and Hadley^21^. In brief, the reaction mixture comprising 8.1% sodium dodecyl sulfate, 20% acetate buffer (pH 3.5), and 0.8% thiobarbituric acid (TBA) was added to 0.2 ml of gastric tissue homogenate for 3 min. Subsequently, the mixture was incubated at 95 °C for 60 min and then left for cooling. After that, the TBA-reactive substance, MDA, was extracted with 1 ml of H_2_O and 2.5 ml of an n-butanol:pyridine mixture (15:1, v/v). The surface organic layer comprising the MDA, which was generated by lipid peroxidation, was read at 532 nm. The absorbance assessed at 532 nm was presented as nM of MDA.

#### Determination of PGE2 formation using enzyme immunoassays

The stomachs mucosa were weighed, crushed by scissors, and then homogenized at 48 °C in a phosphate buffered saline (PBS) buffer. After that, homogenates were centrifuged at 13,400 rpm for 10 min at room temperature. The pure supernatants were served to determine the concentrations of PGE_2_ through a PGE_2_ monoclonal enzyme immunoassay kit (Sigma-Aldrich, Malaysia).

### Histological evaluation of the gastric mucosa

#### Hematoxylin and eosin staining

Small pieces of the stomach wall were fixed using 10% buffered formalin for 18 h at 4 °C and then immersed in paraffin wax. Subsequently, sections of the stomach were prepared by the microtome at a thickness of 5 μm, and stained with Hematoxylin and Eosin (H & E) for histological assessment.

#### Study of mucosal glycoproteins

Sections of 5 μm thickness from the gastric glandular part were stained with Periodic acid Schiff (PAS) stain to detect the mucus secretion and to assess the variations in both acidic and basic glycoproteins^22^.

#### Immunohistochemical staining

The immunohistochemical technique was conducted using (Dako cytomation, USA). Briefly, the tissue section slides were placed in a hot-air oven for 25 min at 60 °C (Venticell, MMM, Einrichtungen, Germany). De-paraffinization of the tissue sections was done using xylene and graded alcohol. After that, slides were boiled in antigen retrieval solution and then incubated with biotinylated primary antibodies of heat shock protein 70 (Hsp70) (1:500) and Bcl-2-associated protein x (Bax) (1:200) for 15 min. Subsequently, streptavidin conjugated to horseradish peroxidase was added to the slides and then incubated for 15 min. Further incubation for 5 min was done after adding DAB-substrate-chromagen to the slides. Finally, slides were immersed in hematoxylin for 5 sec, washed with distilled water and dipped in weak ammonia (0.037 mol/L) 10 times. Positive results of the immunohistochemical staining can be observed as brown areas under a light microscope.

#### Statistical analysis

All the results were presented as mean ± S.E.M. The data were analyzed using one-way ANOVA followed by Tukey’s post hoc test for multiple comparison using SPSS 18 (Statistical Package for the Social Sciences) software. The probability of p < 0.05 was considered statistically significant.

## Results

### Acute toxicity study

Fourteen days after the intragastric administration of MDLA at 2 different concentrations, there were no behavioral alterations and death was noticed. This was confirmed by the histopathological evaluations for the liver and kidney as well as the serum biochemistry results in which no indications of toxicity were noticed after intragastric administration of the 2 concentrations of MDLA (Fig. 2 and Table 2). These outcomes revealed that MDLA up to an intragastric concentration of 1000 mg/kg was not-toxic in rats.

### Gross evaluation of gastric lesions and changes in gastric wall mucus

The protective effect of MDLA against acidified ethanol (HCl/Ethanol) induced gastric ulceration is presented in Table 3. Our findings revealed that rats pre-treated with omeprazole or MDLA before intragastric administration of acidified ethanol (HCl/Ethanol) (groups 3–5) had considerably decreased areas of stomach ulcerations, as displayed in Table 3. The intragastric administration of acidified ethanol (HCl/Ethanol) resulted in hemorrhagic streaks in the gastric mucosa. In contrast, in a concentration-dependent manner, MDLA considerably inhibited the elongated streak of hemorrhages prompted via acidified ethanol (HCl/Ethanol) and clearly diminished the stomach mucosal injury. In addition, flattening of the gastric mucosal folds was noticed. The results showed that MDLA in a concentration-dependent manner considerably flattened the stomach mucosal folds (Fig. 3). Moreover, the stomach pH and gastric wall mucus were evaluated. Pretreatment with MDLA or omeprazole significantly raised the stomach pH and the gastric wall mucus compared to the animals pretreated with acidified ethanol (HCl/Ethanol) (Table 3).

### Effect of MDLA on measurements of SOD, MDA and PGE_2_

The effect of MDLA on the measurements of SOD, MDA and PGE_2_ is presented in Fig. 4. The levels of SOD and PGE_2_ were significantly reduced in the group pretreated with acidified ethanol (HCl/Ethanol). However, the groups that received MDLA or omeprazole showed a significant increase in the levels of SOD and PGE_2._ In contrast, the administration of acidified ethanol (HCl/Ethanol) to the rats caused a significant increase in their MDA measurements, whereas the intragastric dosage of MDLA or omeprazole significantly reduced their MDA measurements.

### Histological evaluation of gastric lesions

Histological analyses of the gastric slides for group 2 exhibited severe harm of the gastric mucosa with necrotic lesions penetrating deeply into the mucosa. In addition, histopathological signs, such as extensive edema and leukocyte infiltration of the submucosal layer, were also detected in this group (Fig. 5). However, the rats in groups 4 and 5 displayed less mucosal injury in comparison to the animals in group 2. The reduced mucosal damage was evidenced by the decrease or non-existence of the ulcer area, edema and leukocyte infiltration (Fig. 5).

### Periodic acid Schiff (PAS) of mucosal glycoproteins

As displayed in Fig. 5, pretreatment with acidified ethanol (HCl/Ethanol) resulted in reduced mucus secretion, as demonstrated by the smaller amount of magenta color in the stomach tissue. In contrast, pretreatment with MDLA or omeprazole caused an increase in the intensity of the magenta color.

### Immunohistochemistry

The immunohistochemical results demonstrated that animal groups administered with MDLA or omeprazole had a large immunostained area of Hsp70 protein. Conversely, the immunostained area of this protein in the groups administrated with acidified ethanol (HCl/Ethanol) was smaller compared to the groups dosed with MDLA or omeprazole (Fig. 6). In addition, the immunohistochemical staining of the Bax protein from the animals pretreated with MDLA or omeprazole confirmed down-regulation of this protein, while ingestion of the acidified ethanol (HCl/Ethanol) resulted in over-regulation of Bax (Fig. 6).

## Discussion

The current report is an endeavor to study the anti-ulcerogenic activity of the new Mn (II) complex with Schiff base derived from 4-dimethylaminobenzaldehyde with L-asparagine against HCl/Ethanol-induced acute gastric ulcerations in rats. The usage of Schiff bases encompassing hetero atoms for the purpose of protection and healing of human ailments is progressing and attracting extraordinary consideration because of their health-promoting properties^23^,^24^.

An elemental analysis data of the Schiff base complex Table (1) show the formation of a 1:1 [M: L] ratio. It was found that the theoretical values are in a good agreement with those identified. The purity of the Schiff base complex was tested using the TLC technique and (C, H and N) elemental analysis. The IR spectrum of the L-asparagine Schiff base complex, which exhibits bands at 1576 cm^−1^, is attributed to ν(C = N) of the azomethine; the changing of this band indicates its involvement in complexation with the metal ions. The infrared spectral results of the same Schiff base complexes show a band at 1603/cm suggesting the existence of the (COO-) group in the L-asparagine compound. This band appears in a higher region compared to its original position in the free ligand 1506 cm^1^. The same spectrum exhibits a broad band at 3466 cm^−1^, which is attributed to the presence of water molecules during the complex formation. The appearance of new bands at 510 cm^−1^ and 596 cm^−1^, which are attributed to ν(M–N) and ν(M–O) vibrations, confirm the involvement of the nitrogen and oxygen atoms in coordination with metal ions. The absorption band at 315 nm (10500 cm^−1^) is attributed to the 2A2g→2T1g transition. The intensity of the band indicates the presence of an octahedral geometry for the Mn (II)-Schiff base complex. Also, the 1H-NMR spectrum of the ligand shows the following characteristic chemical shifts (DMSO as a solvent): the singlet signal at 8.45 δ ppm corresponds to the hydroxyl proton and peak at 7.9 δ ppm attribution of the proton of the azomethyne proton (CH = N−), and shows an aromatic benzene ring at 7.5–7.2 δ ppm and peak at 2.4 δ ppm attribution of the (CH3)2N. The absence of –OH proton is due to complexation. There is an appreciable change in all the other signals in this complex.

The process of drug development requires preclinical evaluation and toxicity studies to ensure the safety of this drug^25^. The current study did not reveal any marks of toxicity or mortality within the two-week period of the experiment. In addition, the histopathological assessment for the liver and kidney, and biochemical analysis of the serum did not display any variance relative to the control group, thereby demonstrating the safety of MDLA when administered intragastrically up to 1 g/kg.

Gastric mucus has a significant role in the protection of the stomach against irritating substances, such as HCl and ethanol, through which the stomach releases a continuous transparent mucus like gel. This gel acts as a defensive barrier to cover the whole gastric mucosa, and, subsequently, sustains the basophilic pH of the mucosal surface. The gastric ulceration disruption of the mucosal defenses may cause severe damage as well as affect the digestive acids^26^. The important principles to evaluate the condition of the mucosal barrier against the aggressive attack of hydrochloric acid and pepsin are the quality and quantity of stomach mucus secretion^27^.

It was reported that an increase in level of gastric wall mucus released by the gastric mucosal cells prevents the ulceration by performing as an efficient fence against the back diffusion of hydrogen ions, thereby ameliorating the storing of digestive acids, and, consequently, decreasing the gastric wall friction upon peristalsis^28^. The outcome from this study shows that pretreatment with MDLA is able to increase the quantity of mucus production, suggesting that the protective effect of MDLA might be attributed to the capability of this compound to enhance the gastric mucosal defense action.

It is known that mucin-type glycoprotein are one of the basic components of the gastric mucus (mucin), which can be detected using the Alcian blue binding assay^19^. Alcian blue dye has the ability to connect with negatively charged substances. According to the results, the upsurge in bound Alcian blue signifies the protective intragastric action of MDLA that can be attributed to the resultant complexes from the reaction between MDLA and the mucus. These complexes act as a barrier against the necrotizing materials introduced in the gastric.

Mucus and bicarbonate secretion play an important role in the process of ulcer prevention. Their significance comes from their efficacy to form a mucus/bicarbonate barrier that is able to protect newly formed cells against acid and peptic damage^29^. Using the PAS staining technique, the stomach regions that secreted mucopolysaccharides seem to have the magenta color. Our findings demonstrate that intragastric administration of MDLA causes intense secretion of mucus in the gastric glands.

The pathogenesis of acidified ethanol (HCl/Ethanol) against gastric tissue probably occurs due to various mechanisms, such as cytokines, lipid peroxidation, generation of reactive oxygen species, oxidative damage, alterations in permeability, and depolarization of the mitochondrial membrane prior to cell death. The ingestion of acidified ethanol (HCl/Ethanol) produces longitudinal hemorrhagic injuries, acute tissue edema, cellular mucosal exfoliation, time-dependent infiltration by inflammatory cell, and epithelial friability in the gastric, which have similar features to lesions resulting from alcohol abuse^30^. The results of the current report show that intragastric administration of MDLA significantly decrease the incidence and acuteness of gastric injuries, and, consequently, reduce the ulcer index (UI) thereby demonstrating the gastroprotictive effect of this compound.

Omeprazole is a proton pump inhibitor (PPI) that suppresses gastric acid secretion via inhibiting hydrogen/potassium ATPase enzyme system in the gastric parietal cells surface that results in pump inactivation. Omeprazole is the common drug of choice used in the treatment of peptic ulcer disease and heartburn^31^. The stimulation and infiltration of neutrophils seem to be engaged in the early events which form the injuries. According to Al Batran *et al.*^32^, the decline in the neutrophil infiltration in the ulcerated mucosa of the stomach triggers the protection of gastric ulcerations in rats. Our investigation shows that the pretreatment of rats with MDLA significantly prevents the gastric tissue and suppresses leukocyte infiltration of the gastric wall.

There are considerable evidences linking the changes in gastric motility and the prevention of gastric lesions that have been induced experimentally. In addition, the resulting flattening of the gastric folds may contribute to ulcer prevention by expanding the mucosal area exposed to necrotizing substances and thus diminish the volume of the gastric irritants on the rugal crest^32^,^33^. Consistent with such evidence, flattening of the mucosal folds was observed in the groups pretreated with MDLA, which indicates that the gastroprotective effect of MDLA might be due to a reduction of the gastric movement.

It is well known that acidified ethanol (HCl/Ethanol) is capable of inducing mucosal damage in the animal models through the triggering of reactive oxygen metabolites^34^. As a response to the accumulation of free radicals, cellular antioxidant enzymes, such as catalase and superoxide dismutase, which are considered as a first defense line against cellular oxidative damage, are released^35^. Superoxide dismutase (SOD) transforms superoxide (O_2_^−^) to hydrogen peroxide (H_2_O_2_)^35^. Whereas, malonaldehyde (MDA) is the final product of lipid peroxidation and is utilized as an indicator of lipid peroxidation^36^. Our experimental results show a significant reduction in the MDA levels followed by a significant increase in the SOD levels after the intragastric administration of MDLA.

Prostaglandin E_2_ (PGE_2_) plays a vital part in the regulation of gastric secretion and motility^36^. In addition, stress is a causative factor of the deactivation of prostaglandin synthetase enzyme that leads to a reduction in the production of prostaglandin, the main defensive mediator against gastric lesions. In the present study, the mucosal level of PGE_2_ shows a significant increase in the biosynthesis of PGE_2_ after pretreatment with MDLA, which suggests that the gastroprotective effect of MDLA may be partially attributed to PGE_2_.

Heat shock protein (Hsp70) is a potential therapeutic target to protect the gastric mucosa from oxidative injury. The inhibition of Hsp70 provoked gastric cellular damage induced by acidified ethanol (HCl/Ethanol), as reported previously in many studies^37^,^38^. In this study, the gastric tissues that received MDLA revealed over expression of Hsp70 proteins, thus suggesting that the up-regulation of Hsp70 might play an important role in the gastroprotective of MDLA by reducing the reactive oxygen species-mediated gastric oxidative stress.

Considerable evidence indicates the role of apoptosis (programmed cell death) in gastric ulceration^3^. In the normal physiological status, stomach mucosal layer always be in balance between the cell death and cell renewal process. Gastric injuries increase when there is a rise in cell death and/or suppression of cell production^3^. It was evidenced that acidified ethanol (HCl/Ethanol) induced gastric damage by accelerating apoptosis^39^. Bcl-2 family proteins have a fundamental part in controlling apoptosis, and up to 14 members of Bcl-2 family have been identified. The first category of this family is the pro-apoptotic proteins, such as Bax, Bak, and Bcl-Xs, while the second category comprises the anti-aopoptotic proteins, such as Bcl-2, Bcl-XL, and Mcl-1^39^. In this study, the effect of MDLA against apoptosis of stomach tissue was determined through Bax expression in the gastric tissue after acidified ethanol (HCl/Ethanol)-induced gastric ulcer. The outcomes displayed that treatment with MDLA exhibited a down regulation of the Bax protein expression in the gastric mucosal tissue as shown by immunohistochemical staining. This result suggests that MDLA effectively inhibits acidified ethanol (HCl/Ethanol) ulceration through its anti-apoptotic properties.

## Conclusion

Toxicity investigations affirmed the safety of MDLA up to 1 g/kg. In a concentration-dependent manner, MDLA considerably presented gastroprotective activity against acidified ethanol (HCl/Ethanol)-induced gastric injuries in Sprague Dawley rats. The antiulcerogenic efficacy of MDLA could be related to the participation of mucus, free radical scavenging capacity and stimulation of the cellular antioxidant mechanism by increasing the gastric SOD level and decreasing the lipid peroxidation addition to the upregulation of Hsp70 protein. Moreover, MDLA demonstrated a significant reduction in the pro-apoptotic protein of Bax. The current report warrants further investigation on MDLA as a promising gastroprotective candidate.

## Additional Information

**How to cite this article**: Ibrahim, M. Y. *et al.* Acute Toxicity and Gastroprotection Studies of a New Schiff Base Derived Manganese (II) Complex against HCl/Ethanol-Induced Gastric Ulcerations in Rats. *Sci. Rep.* **6**, 26819; doi: 10.1038/srep26819 (2016).

## Figures and Tables

**Figure 1:** Chemical structure of MDLA [Mn L (H_2_O) _3_(OH)].

**Figure 2:** Effect of MDLA on histological sections of the liver and kidney in rats. (**A,B**) Rats treated with vehicle. (**C,D**) Rats treated with 500 mg/kg of MDLA. (**E**,**F**) Rats treated with 1000 mg/kg of MDLA. There is no significant difference in the architecture of the livers and kidneys between the treated and control groups (H&E stain, 20× magnifications).

**Figure 3:** Macroscopic appearance of the gastric mucosa in HCl/Ethanol induced gastric ulcer in rats. (G1) Group 1 has no injury to the gastric mucosa. (G2) Group 2 have severe injuries in the gastric mucosa. HCl/Ethanol produced extensive visible hemorrhagic necrosis of the gastric mucosa. (G3) Rats in group 3 pretreated with omeprazole have mild injuries to the gastric mucosa, comparing to the injuries observed in group 2. (G4) Rats in group 4 have moderate injuries in the gastric mucosa. MDLA reduces the formation of gastric lesions induced by HCl/Ethanol. (G5) Rats in group 5 have mild injuries in the gastric mucosa. Black arrows show the location of the lesions inside the gastric mucosa.

**Figure 4:** The effect of MDLA on MDA level (μmol/g protein), SOD activity (U/g protein) and PGE2 (pg/mg protein) in gastric mucosal homogenate in rats. MDLA increased the PGE2 and SOD, and decreased the level of lipid peroxidation (MDA) in the pre-treated groups. All values are expressed as mean ± standard error mean, the mean difference is significant at (*p < 0.05) level compared to CMC (Control). Data were analyzed using one way ANOVA using SPSS 18.

**Figure 5:** The histological effect of MDLA on gastric mucosal (H&E) and gastric tissue glycoprotein-PAS staining in HCl/Ethanol induced gastric ulcer in rats. (G1) (Normal control group); Rats in group 1 have no disruption of the surface epithelium. (G2) (Ulcer control group); Rats in group 2 have severe disruption of the surface epithelium (red arrow) and necrotic lesions that penetrate deeply into the mucosa (white arrow). Extensive edema of the submucosal layer (yellow arrow) and leukocyte infiltration are present (yellow arrow). (G3) (omeprazole); Group 3 has mild disruption of the surface epithelium, and there is a submucosal edema and leucocyte infiltration (blue arrow). (G4) (MDLA 10 mg/kg); Group 4 has moderate disruption of the surface epithelium with edema and leucocytes infiltration of the submucosal layer (blue arrow). (G5) (MDLA 20 mg/kg); Rats in group 5 showed a mild disruption of the surface epithelium with edema and leucocyte infiltrationin submucosal layer (blue arrow) (H&E staining, 20×). The gastric mucosa in animals pretreated with MDLA or omeprazole (group 3–5) displayed increased PAS staining intensity compared to the rats in group 2, indicating an increase in the glycoprotein content of gastric mucosa in pretreated rats (blue arrows) (PAS stain 20×).

**Figure 6:** Effects MDLA on the immunohistochemistry analysis of expression of Hsp70 and Bax proteins in HCl/Ethanol induced gastric ulcer in rats. Normal control group (G1), ulcer control group (G2), omeprazole-treated group 20 mg/kg (G3), rats receiving 500 mg/kg of MDLA (G 4), and rats receiving 1000 mg/kg of MDLA (G5). Immunohistochemistry staining of Hsp70 shows over-expression of Hsp70 protein in the experimental groups (G3, G4 and G5). Meanwhile, Bax protein expression was downregulated in the experimental groups (G3, G4 and G5) (magnification 20×).

**Table 1:** Elemental analysis and spectral characterization for the ligand and its metal complex.

Ligand Elemental Analysis	Analytical Calculated: C, 64.07; H, 6.79; N, 13.59.
Found: C, 64.02; H, 6.75; N, 13.53.	
IR (KBr)v	(OH), 3397; v(C = N), 1576; v(C OO-)1506.
UV-Vis (DMSO), λmax (€ Mol^−1^cm^−1^):	280 nm (9333, (**π→π**); 343 nm (11433, (nπ*)
1H-NMR (DMSO-d6)	2.49 (s, 6H, CH3), 7.50–7.20 (4H, ArH), 7.94 (s, 1H, azomethine), 8.45 (s, 1H, OH)
Complex Elemental Analysis	Analytical Calculated: C, 39.88; H, 6.04; N, 8.46
Found: C, 39.54; H, 5.95; N, 8.40.	
IR (ATR cm21)	v(OH), 3466; v(C = N), 1659; v(C OO-), 1603 v(M-N), 510 v(M-O)596.
UV-Vis (DMSO)	295 (π→π*); 315 (n→π*); 500 (d → d*).
1H-NMR (DMSO-d6)2.30 (s, 6 H, CH3), 7.30–6.76 (4 H, ArH), 8.5 (s, 1 H, azmthen)	

**Table 2:** Serum biochemical data for male and female rats intragastrically administered. MDLA for 14 days.

Parameter	Sex	Normal 0.5% CMC	MDLA 500 mg/kg	MDLA 1000 mg/kg
sodium mmol/L	Male	151.75 ± 0.48	150.00 ± 3.14	152.00 ± 3.7
	Female	151.3 + 0.63	152.8 ± 2.3	153.8 ± 1.44
potassium mmol/L	Male	4.91 ± 0.15	5.08 ± 0.43	5.45 ± 0.9
	Female	5.34 + 0.10	5.7 ± 0.0.3	6.0 ± 0.4
chloride mmol/L	Male	102.75 ± 0.75	101.50 ± 7.1	99.50 ± 6.7
	Female	100.2 + 1.7	99.3 ± 9.76	101.8 ± 7.5
carbon dioxide mmol/L	Male	14.52 ± 0.78	14.02 ± 0.83	15.05 ± 1.4
	Female	13.6 + 0.87	14.7 ± 0.5	14.8 ± 1.3
anion gap mmol/L	Male	25.00 ± 0.41	26.25 ± 2.25	27.50 ± 2.22
	Female	28.8 + 0.48	27.8 ± 2.1	29.0 ± 2.7
urea nitrogen mmol/L	Male	9.73 ± 0.55	10.52 ± 1.82	11.82 ± 1.67
	Female	10.2 + 0.43	11.8 ± 1.4	12.3 ± 1.6
creatinine umol/L	Male	30.50 ± 1.55	31.00 ± 1.63	32.50 ± 2.96
	Female	28.3 + 1.3	28.5 ± 2.6	27.3 ± 2.95
total protein g/L	Male	59.40 ± 2.5	60.00 ± 1.47	59.50 ± 2.8
	Female	60.8 ± 1.75	60.3 ± 2.29	61.3 ± 1.44
albumin g/L	Male	13.70 ± 0.41	13.75 ± 1.25	14.75 ± 0.75
	Female	14.2 ± 0.41	15.0 ± 0.71	15.0 ± 1.1
globulin g/L	Male	49.00 ± 1.96	50.00 ± 1.22	51.50 ± 3.1
	Female	51.7 ± 2.48	52.3 ± 3.57	52.6 ± 1.92
total bilirubin umol/L	Male	3.65 ± 0.25	3.25 ± 0.25	3.0 ± 0.0
	Female	3.2 ± 0.29	3.0 ± 0.00	2.9 ± 0.25
alkaline phosphatase IU/L	Male	87.50 ± 3.57	89.75 ± 5.2	88.75 ± 5.33
	female	96.0 ± 1.87	95.3 ± 5.76	96.00 ± 4.16
alanine aminotransferase IU/L	Male	58.75 ± 1.55	59.75 ± 1.18	60.00 ± 1.58
	Female	61.3 ± 2.75	62.0 ± 1.35	62.3 ± 2.06
Ast IU/L	Male	189.0 ± 5.51	194.8 ± 10.59	196.5 ± 12.6
	Female	191.0 ± 4.26	193.0 ± 3.58	192.8 ± 11.21

Values are expressed as mean ± SEM. There are no significant differences between groups significant value at P < 0.05.

**Table 3:** Effect of MDLA on gastric ulcer area, inhibition percentage and changes in Alcian blue binding capacity in gastric mucosa of rats.

Pre-treatment (5 ml/kg dose)	Ulcer area (mm)^2^	Inhibition (%)	pH	Gastric volume	ABB (mg Alcian blue/g of tissue)
CMC (Vehicle control)*	–	–	7.03 ± 0.00	1.12 ± 0.00	723.76 ± 1.05
CMC (Ulcer control)	972.34 ± 0.97	–	3.02 ± 0.02	0.33 ± 0.00	321.10 ± 0.97
Omeprazole (20 mg/kg)	138.84 ± 0.71*	85.72*	5.62 ± 0.00*	0.98 ± 0.01*	743.52 ± 0.69*
MDLA (10 mg/kg)	422.83 ± 0.72*	56.51*	4.94 ± 0.01*	0.72 ± 0.00*	674.70 ± 0.85*
MDLA (20 mg/kg)	331.25 ± 0.58*	65.93*	5.52 ± 0.01*	0.82 ± 0.00*	705.94 ± 1.13*

Ulcer area and Inhibition: ulcer induced by HCl/Ethanol. Gastric pH, gastric volume and Alcian blue bound (ABB): ulcer induced by Shay ulcer. Rats pre-treated with MDLA had significantly reduced areas of gastric ulcers and pH of gastric content for groups pre-treated with MDLA (10 and 20 mg/kg), respectively. All values are expressed as the mean ± standard error mean, the mean difference is significant at (*p < 0.001) level compared to CMC (Ulcer control). Data were analyzed using One Way ANOVA, using the statistics software and analytical solutions SPSS 18.
